The article "CAIX is a predictor of pathological complete response and is associated with higher survival in locally advanced breast cancer submitted to neoadjuvant chemotherapy" was published in 2019. Journal: BMC Cancer.

# CAIX is a predictor of pathological complete response and is associated with higher survival in locally advanced breast cancer submitted to neoadjuvant chemotherapy

**DOI:** 10.1186/s12885-019-6353-2

**Published:** 2019-12-03

**Authors:** Wilson Eduardo Furlan Matos Alves, Murilo Bonatelli, Rozany Dufloth, Lígia Maria Kerr, Guilherme Freire Angotti Carrara, Ricardo Filipe Alves da Costa, Cristovam Scapulatempo-Neto, Daniel Tiezzi, René Aloísio da Costa Vieira, Céline Pinheiro

**Affiliations:** 1 Nuclear Medicine and Molecular Imaging Department, Barretos Cancer Hospital – Pio XII Foundation, Rua Antenor Duarte Vilela, N° 1331, Barretos, São Paulo 14784-400 Brazil; 2 Molecular Oncology Research Center, Barretos Cancer Hospital, Barretos, São Paulo Brazil; 3 Pathology Department, Barretos Cancer Hospital, Barretos, São Paulo Brazil; 4 Surgery Department, Federal University of Triangulo Mineiro, Uberaba, Minas Gerais Brazil; 5 Research and Teaching Institute, Barretos Cancer Hospital, Barretos, São Paulo Brazil; 6 Barretos School of Health Sciences Dr. Paulo Prata - FACISB, Barretos, São Paulo Brazil; 7 Department of Gynecology and Obstetrics – Breast Disease Division, Faculty of Medicine of Ribeirão Preto, University of São Paulo, Ribreirão Preto, São Paulo Brazil; 8 Department of Mastology and Breast Reconstruction, Barretos Cancer Hospital, Barretos, São Paulo Brazil

**Keywords:** Breast cancer, CAIX, Glycolytic metabolism, Immunohistochemistry, Neoadjuvant chemotherapy, Pathological complete response

## Abstract

**Background:**

Locally advanced breast cancer often undergoes neoadjuvant chemotherapy (NAC), which allows in vivo evaluation of the therapeutic response. The determination of the pathological complete response (pCR) is one way to evaluate the response to neoadjuvant chemotherapy. However, the rate of pCR differs significantly between molecular subtypes and the cause is not yet determined. Recently, the metabolic reprogramming of cancer cells and its implications for tumor growth and dissemination has gained increasing prominence and could contribute to a better understanding of NAC. Thus, this study proposed to evaluate the expression of metabolism-related proteins and its association with pCR and survival rates.

**Methods:**

The expression of monocarboxylate transporters 1 and 4 (MCT1 and MCT4, respectively), cluster of differentiation 147 (CD147), glucose transporter-1 (GLUT1) and carbonic anhydrase IX (CAIX) was analyzed in 196 locally advanced breast cancer samples prior to NAC. The results were associated with clinical-pathological characteristics, occurrence of pCR, disease-free survival (DFS), disease-specific survival (DSS) and overall survival (OS).

**Results:**

The occurrence of pCR was higher in the group of patients whith tumors expressing GLUT1 and CAIX than in the group without expression (27.8% versus 13.1%, *p* = 0.030 and 46.2% versus 13.5%, *p* = 0.007, respectively). Together with regional lymph nodes staging and mitotic staging, CAIX expression was considered an independent predictor of pCR. In addition, CAIX expression was associated with DFS and DSS (*p* = 0.005 and *p* = 0.012, respectively).

**Conclusions:**

CAIX expression was a predictor of pCR and was associated with higher DFS and DSS in locally advanced breast cancer patients subjected to NAC.

## Background

Breast cancer (BC) is one of the most prevalent tumors in the world and the most frequent malignancy in women [1]. In the United States of America, only in 2018, approximately 266,000 new cases and close to 41,000 deaths are expected due to BC [2]. In developing countries such as Brazil, the incidence of BC is lower, but the ratio between mortality and incidence is higher than in developing countries [3, 4] and this is associated with a high number of patients diagnosed at a later stage [5]. Neoadjuvant chemotherapy (NAC) is a therapeutic option for locally advanced tumors allowing early treatment of micrometastatic disease, in vivo evaluation of the therapeutic response, increased conservative surgery rate due to tumor shrinkage and prognostic evaluation based on clinical and pathological responses [6].

Defined as the absence of residual invasive carcinoma after NAC in the breast or lymph nodes, the pathological complete response (pCR) is associated with greater overall survival (OS) and disease-free survival (DFS) [7–9]. However, pCR rate differs significantly between molecular subtypes. Although triple-negative tumors are more aggressive with high relapse rates and unfavorable prognosis, they are more chemosensitive with pCR rates ranging from 45 to 56% [10–12]. Among luminal subtypes, the association between pCR and DFS is observed in luminal B / HER2- but not in luminal A and luminal B / HER2+ [8]. Thus, pCR presents important variations between and within the tumor subgroups and does not seem to be directly related to their clinical characteristics. Thus, it is necessary to know more about other tumor characteristics to better establish the relationship between pathological response and clinical evolution. In this context, information about the metabolic phenotype of cancer cells may provide new insights into factors influencing pathological response and prognosis.

Interest in the metabolic profile of BC has grown after the introduction of Positron Emission Tomography (PET) in clinical practice, which uses a glucose analog fluorine-18 fluorodeoxyglucose (^18^F-FDG) for evaluation of tumor metabolism [13]. It is known that the main energetic pathway in cancer cells is glycolysis and glucose consumption is much higher in tumors than in normal cells [14]. The preferred use of the glycolytic pathway is related to a series of alterations in tumor cells, which include hypoxia, increased expression of proteins related to glycolytic metabolism and acidification of the extracellular environment [14–17]. All these changes in the tumor microenvironment determine the selection of cells with an acid-resistant hyperglycolytic phenotype [16], associated with increased aggressiveness, growth and dissemination of BC [18–20].

Some proteins are essential for the effective control of tumor metabolism, including glucose transporter-1 (GLUT1), the main protein responsible for glucose influx [14]. Proteins related to intracellular pH control and acidification of the extracellular medium, such as carbonic anhydrase IX (CAIX) and monocarboxylate transporters (MCTs), are essential for cellular metabolism control as well [15]. CAIX is related to H^+^ efflux, acting as a catalyst in a reversible carbon dioxide hydration reaction and its expression has been associated with a worse prognosis in several tumors, including BC [14, 17]. The monocarboxylate transporters MCT1 and MCT4, associated with their anchoring protein CD147, have a determinant role in the metabolic reprogramming of cancer cells towards a hyperglycolytic phenotype by promoting the efflux of lactate and pyruvate and, consequently, helping the control of cellular pH, as well as allowing high glycolytic flux [16]. The expression of GLUT1, MCT1, MCT4, and CD147 appears to be associated with increased aggressiveness and lower DFS in BC [19–21].

The aim of this study was to evaluate the expression of MCT1, MCT4, CD147, GLUT1 and CAIX in locally advanced BC submitted to NAC and their relationship with pCR, DFS, disease-specific survival (DSS) and OS.

## Methods

### Patients and clinicopathologic data

This is a retrospective study approved by the local ethics committee. Clinical and anatomopathological data from 328 female patients admitted consecutively to Barretos Cancer Hospital from 2005 to 2011, with locally advanced breast cancer, clinical stage IIb or III, were used. All patients underwent chemotherapy based on a regimen of doxorubicin plus cyclophosphamide, associated with paclitaxel. Exclusion criteria included: (i) cases whose TMA’s tumor samples were not sufficiently representative for evaluation of protein expression; (ii) cases with expression result only for one or two markers; (iii) cases in which clinicopathologic data of interest could not be properly collected from the review of medical records filed at the Barretos Cancer Hospital. After the completion of IHC to evaluate the expression of glycolytic metabolism markers and review of clinicopathological data, the final sample of the study included 196 patients. Of the 132 excluded patients, 19 presented insufficient clinical data on the medical records; 92 did not present representative material in the TMA; and, 21 had expression results for only one or two of the proteins studied.

For all patients, sequential chemotherapy with 4 cycles of doxorubicin 60 mg / m^2^ and cyclophosphamide 600 mg / m^2^ (AC), followed by 4 cycles each 3 weeks or 12 cycles weekly of paclitaxel 175 mg / m^2^ (T) was delivered to all patients. Breast surgery and adjuvant radiotherapy were done after NAC. The patients were evaluated every 6 months in the first 5 years of follow-up and annually thereafter. The total follow-up time was considered from the date of hospital admission (date of the first consultation) to the date of the last follow-up visit. The disease-free survival was determined from the date of surgery to the date of the first recurrence (documented by imaging examination) or the date of the last follow-up visit.

The mean age of patients was 49.6 years (range: 29.8–76.0 years) and the mean of the largest tumor diameter was 6.8 cm (range: 2.0–20.0 cm). For synchronous bilateral tumors (1% of cases), we considered the measurement of the largest tumor. At the end of NAC, 75% of the patients used 4 AC + 4 T, 11.7% of 4 AC + 12 T and 13.3% of another chemotherapy regimen. The mean of the largest tumor diameter after NAC was 2.93 cm (range: 0.0–14.0 cm). The surgical treatment was mastectomy in 79.1% of cases and conservative surgery in the remaining ones. All patients had axillary region surgically approached, with axillary clearance occurring in 98.5% of cases and sentinel lymph node investigation in the others. All clinicopathologic features used in analysis of this study are summarized in Table 1.

**Table 1:** Clinicopathologic characteristics of BC samples, before NAC, for all patients included (*n* = 196^a^)

Characteristics	Categories	n	%
TNM - T	T1	2	1.0
	T2	17	8.7
	T3	102	52.0
	T4	75	38.3
TNM - N	N0	22	11.2
	N1	116	59.2
	N2	51	26.0
	N3	7	3.6
TNM - M	M0	196	100.0
Histological type	Invasive no special type (NST)	169	86.2
	Others	27	13.8
Nottingham histological grade	I	16	8.2
	II	84	42.9
	III	96	49.0
Tubule formation	> 75%	4	2.0
	10–75%	16	8.2
	< 10%	176	89.8
Mitotic rate	1	76	38.8
	2	59	30.1
	3	61	31.1
Nuclear grade	G1	12	6.1
	G2	50	25.5
	G3	134	68.4
Necrosis	Absent	121	61.7
	Present	75	38.3
Lymphatic invasion	Absent	156	80.4
	Present	38	19.6
Inflammatory infiltrate	Absent	44	22.4
	Present	152	77.6
Ki67	< 14%	25	12.8
	≥ 14%	171	87.2
Estrogen receptor	Negative	64	32.7
	Positive	132	67.3
Progesterone receptor	Negative	85	43.4
	Positive	111	56.6
HER2 overexpression	Negative	129	65.8
	Positive	67	34.2
Subtype	Luminal A	22	11.2
	Luminal B/HER2 -	77	39.3
	Luminal B/HER2 +	46	23.5
	HER2	20	10.2
	Triple-negative	31	15.8

(^a^) Excepted at Lymphatic invasion, where *n* = 194

The median follow-up time was 73.9 months (time range, 10.6–125.1 months) and the median DFS was 55.9 months (time range, 1–113 months). Metastatic tumor recurrence was observed in 91 (46.4%) patients, and locoregional recurrence (isolated or simultaneous to distance recurrence) was observed in 42 (21.4%). The most compromised sites of distance metastasis were bones (56 cases - 28.6%) and lungs (40 cases - 20.4%).

The pathological data related to BC of each patient before NAC were obtained from biopsy samples and the tumor samples were organized into tissue microarray (TMA). The TMA was made after histological review by a pathologist. Tumor samples were represented in the TMA by 1.5 mm diameter cores. Several clinicopathologic characteristics were recorded as follow: AJCC TNM stage (7th edition), histological type (invasive no special type –NST - or others), Nottingham histological grade (I – III), tubule formation (> 75%, 10–75% or <  10%), mitotic rate (1–3), nuclear grade (G1 – G3), necrosis (absent or present), lymphatic invasion (absent or present), Inflammatory infiltrate (absent or present), Ki67 expression (< 14% or ≥ 14%), estrogen and progesterone receptors expressions (negative or positive), HER2 overexpression (negative or positive) and immunohistochemical subtype (luminal A, luminal B / HER2-, luminal B / HER2+, HER2 and triple-negative). The luminal A subtype presents estrogen and progesterone receptors expressions and Ki67 <  14%; the luminal B subtypes have estrogen and progesterone receptors expressions and Ki67 ≥ 14% with or without HER2 overexpression; the HER2 presents only HER2 overexpression; and triple-negative subtype does not present estrogen and progesterone receptors expressions neither HER2 overexpression.

pCR evaluation was performed after NAC in samples obtained from the analysis of the surgical specimen. The pCR was classified as present or absent based on the criteria of the National Surgical Adjuvant Breast and Bowel Project (NSABP) [22]. The percentage of pCR in this study was 16.3%, with 9.1% in luminal A, 9.1% in luminal B / HER2-, 26.1% in luminal B / HER2+, 25.0% in HER2 and 19.4% in triple-negative.

### Immunohistochemistry

The immunohistochemical reactions were performed in the TMA sections according to the avidin-biotin-peroxidase complex principle, using the UltraVision™ LP Detection System (Thermo Scientific™ Lab Vision™) kits for MCT1 and CD147 proteins and Advance™ HRP (Dako®) for the others, following the indications of the manufacturers and according to the details previously described by the group [23]. First, the TMA sections were deparaffinized and hydrated followed by antigen retrieval with the use of EDTA buffer (1 mM, pH 8) for CD147 or citrate (0.01 M, pH 6) to the other proteins in controlled heating (98 °C) for 20 min.

For MCT1 detection, sections were incubated with rabbit polyclonal antibody (AB3538P Chemicon International®), diluted 1:400, overnight, and oral cavity squamous cell carcinoma was used as positive control. MCT4 detection was performed with goat polyclonal antibody (sc-50,329 Santa Cruz Biotechnology®), diluted 1:200, for 2 h, and oral squamous cell carcinoma was used as positive control. CD147 reaction was done with mouse monoclonal antibody (clone 1.BB.218, sc-71,038 Santa Cruz Biotechnology®), diluted 1:500, overnight, and normal colon was used as positive control. For GLUT1, rabbit polyclonal antibody (ab15309–500 AbCam Plc®) was diluted 1:200, incubated for 2 h, and placenta used as positive control. CAIX was detected with rabbit polyclonal antibody (ab15086 AbCam Plc®), diluted 1:200, for 2 h, and normal gastric tissue was used as positive control. Finally, slides were counterstained with hematoxylin and permanently mounted.

The IHC reactions were assessed by two observers, who scored the sections semiquantitatively in relation to the positive control as previously described [17, 24]: 0, 0% of immunoreactive cells; 1, < 5% of immunoreactive cells; 2, 5–50% of immunoreactive cells; and 3, > 50% of immunoreactive cells. Also, intensity of staining was scored as 0, negative; 1, weak; 2, intermediate; and 3, strong. Final immunoreactivity score was defined as the sum of both parameters (extent and intensity) and grouped as negative (score 0 and 2) and positive (3–6) [17, 24]. Discordant results were discussed by the same two observers at a double-head microscope to reach a final score. The two observers analyzed membrane and cytoplasmic expressions of the metabolism-related proteins in all samples. However, due to the functional aspect, only membrane expression was considered in the statistical analysis.

### Statistical analysis

The results obtained were analyzed using the statistical software IBM®-SPSS (version 20). All comparisons were examined for statistical significance using Pearson chi-square test (χ2) or Fisher’s exact test, as appropriate. Multivariate logistic regression was performed for variables with *p*-value < 0.20 at univariate regression.

OS, DSS and DFS curves were plotted using Kaplan-Meier method. Log-rank test was performed to compare survival curves for all characteristics. The characteristics that showed p-value < 0.20 at log-rank test were selected for the Cox proportional hazards regression model. For all statistical analyses, a significance level of 5% (p-value < 0.05) was adopted.

## Results

### Expression of proteins related to glycolytic metabolism

The membrane and cytoplasmic expressions of metabolism-related proteins can be observed at Fig. 1. Considering only membrane analysis, MCT1, MCT4, CD147, GLUT1 and CAIX expression in the sample was 6.5% (12/174), 9.4% (17/163), 2.2% (4/181), 19% (36/153) and 7.4% (13/163), respectively.

**Fig. 1:** Representative images of the immunohistochemical findings (membrane and citoplasmatic expressions) for the different metabolism-related proteins in breast cancer samples. **a** MCT1; **b** MCT4; **c** CD147; **d** GLUT1; **e** CAIX

The association between metabolism-related proteins and clinicopathologic characteristics was also evaluated (Additional file 1: Table S1). For MCT1 expression, there was a statistically significant association with absence of estrogen receptor (ER) (*p* = 0.042) and progesterone receptor (PR) (*p* = 0.032), mitotic rate 3 (*p* = 0.038) and Nottingham histological grade III (*p* = 0.001). Regarding MCT4 expression, there were statistically significant associations with primary tumor staging (TNM - T) (*p* = 0.018), regional lymph nodes staging (TNM - N) (*p* = 0.048) and necrosis occurrence (*p* = 0.019). When the association of CD147 with clinical and pathological characteristics was analyzed, there was association with regional lymph nodes staging (TNM - N) (*p* = 0.017), triple-negative subtype (*p* = 0.030) and absence of PR (*p* = 0.041). GLUT1 expression was a significantly associated with primary tumor staging (TNM - T) (*p* = 0.020), regional lymph nodes staging (TNM - N) (p = 0.001), nuclear grade G3 (*p* = 0.031) and presence of necrosis (*p* = 0.013). Regarding CAIX expression, there was association with absence of ER (p = 0.019) and PR (*p* = 0.011), nuclear grade G3 (*p* = 0.007) and presence of necrosis (*p* = 0.019).

### Protein expression and clinical and pathological characteristics and their association with pCR

As observed in Table 2, at univariate analysis, characteristics as age <  50 years old, advanced regional lymph nodes staging (TNM-N), HER2 overexpression and GLUT1 and CAIX expressions were associated with pCR. At this same analysis, estrogen receptor expression and mitotic rate 3 occurrence also demonstrated a statistic association, however as negative predictors of pCR.

**Table 2:** Association of clinicopathologic characteristics and proteins related to glycolytic metabolism with pathological complete response (pCR) – univariate and multivariate analysis

Characteristics	Categories	Univariate analysis		Multivariate analysis	
		*Odds Ratio* (95% CI)	*p*	Odds Ratio (95% CI)	*p*
Age (years)	≥ 50	Ref		Ref	
	< 50	2.683 (1.171–6.149)	**0.020**	2.631 (0.856–8.087)	0.091
Histological type	Invasive NST	Ref		Ref	
	Others	0.371 (0.083–1.650)	0.193	0.723(0.114–4.605)	0.731
TNM - T	T1 + T2	Ref		–	
	T3 + T4	1.323 (0.545–3.211)	0.536	–	
TNM - N	N0 + N1	Ref		Ref	
	N2 + N3	3.436 (1.147–10.293)	**0.027**	0.182 (0.038–0.887)	**0.035**
Subtype	Luminal A	Ref		Ref	
	Luminal B/HER2 -	1.000 (0.192–5.197)	1.000	0.458 (0.049–4.311)	0.494
	Luminal B/HER2 +	3.529 (0.716–17.404)	0.121	2.029 (0.067–61.316)	0.684
	HER2	3.333 (0.567–19.593)	0.183	0.647 (0.016–26.726)	0.818
	Triple-negative	2.400 (0.436–13.202)	0.314	0.183 (0.011–2.926)	0.230
Estrogen receptor	Negative	Ref		Ref	
	Positive	0.354 (0.164–0.767)	**0.008**	0.254 (0.041–1.552)	0.138
Progesterone receptor	Negative	Ref		–	
	Positive	1.185 (0.554–2.534)	0.662	–	
HER2 overexpression	Negative	Ref		Ref	
	Positive	2.584 (1.197–5.580)	**0.016**	0.922 (0.057–14.873)	0.954
Ki 67	< 14%	Ref		–	
	≥ 14%	2.447 (0.547–10.940)	0.242	–	
Tubule formation	≥ 10%	Ref		–	
	< 10%	1.118 (0.308–4.063)	0.866	–	
Mitotic rate	1 + 2	Ref		Ref	
	3	0.324 (0.149–0.703)	**0.004**	4.899 (1.439–16.673)	**0.011**
Nuclear grade	G1 + G2	Ref		Ref	
	G3	1.802 (0.734–4.426)	0.199	0.598 (0.140–2.546)	0.487
Nottingham histological grade	G1 + G2	Ref		–	
	G3	1.651 (0.765–3.564)	0.201	–	
Necrosis	Absent	Ref		Ref	
	Present	2.071 (0.964–4.449)	0.062	1.186 (0.3335–4.192)	0.792
Inflammatory infiltrate	Absent	Ref		Ref	
	Present	2.258 (0.747–6.829)	0.149	0.740 (0.188–2.916)	0.667
Lymphatic invasion	Absent	Ref		–	
	Present	0.538 (0.177–1.638)	0.275	–	
MCT1	Negative	Ref		–	
	Positive	0.436 (0.054–3.509)	0.436	–	
MCT4	Negative	Ref		–	
	Positive	0.736 (0.158–3.418)	0.696	–	
CD147	Negative	Ref		–	
	Positive	1.747 (0.176–17.387)	0.634	–	
GLUT1	Negative	Ref		Ref	
	Positive	2.558 (1.074–6.091)	**0.034**	3.166 (0.882–11.360)	0.077
CAIX	Negative	Ref		Ref	
	Positive	5.494 (1.689–17.866)	**0.005**	6.221 (1.148–33.706)	**0.034**

*NST* No Special Type, *Ref* Reference. Significant values are shown in bold

When logistic regression (multivariate analysis) was performed, regional lymph nodes staging (TNM-N), mitotic rate and CAIX expression were considered independent pCR predictors. It is interesting to note that TNM-N and mitosis rate have reversed their association with pCR and only CAIX expression has remained as independent positive predictor of pCR.

### Survival analysis

The association of proteins related to glycolytic metabolism with DFS, DSS, and OS is observed in Table 3, where percentages of patients free of events are showed after 24, 60 and 120 months. Only CAIX expression was associated with DFS and DSS, with *p* = 0.005 and *p* = 0.012, respectively (Fig. 2). Cox regression was performed and none of the proteins related to glycolytic metabolism was considered an independent predictor of survival (Additional file 2: Table S2).

**Table 3:** Percentage of free-events patients over months when associated the expression of proteins related to glycolytic metabolism with survivals (univariate analysis)

Characteristics	Categories	Cases (n)	DFS				DSS				OS			
			24 mo	60 mo	120 mo	*p*	24 mo	60 mo	120 mo	*p*	24 mo	60 mo	120 mo	*p*
MCT1	Negative	174	86.8	68.7	19.5	0.136	91.4	68.6	55.4	0.361	91.4	66.6	51.8	0.507
	Positive	12	91.7	83.3	41.7		91.7	83.3	41.7		91.7	83.3	31.3	
MCT4	Negative	163	85.7	66.6	22.0	0.259	90.7	68.7	49.2	0.982	89.6	66.7	45.7	0.364
	Positive	17	88.2	57.8	28.9		88.2	63.5	63.5		88.2	52.9	45.4	
CD147	Negative	181	86.7	66.4	20.5	0.072	90.6	68.2	48.9	0.374	90.6	67.3	45.8	0.085
	Positive	4	75.0	25.0	25.0		75.0	50.0	50.0		75.0	25.0	25.0	
GLUT1	Negative	153	89.4	66.9	20.5	0.683	92.1	69.2	47.2	0.567	90.8	66.6	43.4	0.584
	Positive	36	83.3	66.7	37.7		91.7	69.2	65.2		91.7	66.7	58.8	
CAIX	Negative	163	84.6	66.1	18.3	**0.005**	89.6	66.0	45.5	**0.012**	89.6	64.9	42.9	0.143
	Positive	13	100.0	100.0	100.0		100.0	100.0	100.0		92.3	84.6	75.2	

*DFS* Disease-free survival, *DSS* Disease-specific survival, *OS* Overall survival, *mo* Months. Significant values are shown in bold

**Fig. 2:** Disease-free survival curve (**a**) and disease-specific survival curve (**b**) of groups with and without CAIX expression. In the curves, DFS and DSS were higher in patients with tumors that expressed CAIX than in those who did not express CAIX (log-rank, *p* = 0.005 and *p* = 0.012, respectively)

## Discussion

The metabolic reprogramming of cancer cells and its implications for tumor growth and dissemination has gained increasing prominence and could contribute to a better understanding of NAC response. Some proteins like glucose tranporters and monocarboxilate transporters are essential for metabolic control and have been characterized as predictors of response and prognostic factors. Thus, this study evaluated the expression of MCT1, MCT4, CD147, GLUT1 and CAIX in locally advanced BC submitted to NAC and their relationship with pCR, DFS, DSS and OS. Unexepectedly, CAIX expression has been showed as predictor of pCR and was associated with higher DFS and DSS in patients with locally advanced breast cancer treated by NAC using AC-T.

The present study evaluated a cohort of patients with breast cancer at stages IIb and III treated with NAC, whose tumor size was greater than 5.0 cm in most of the cases. Moreover, there was a long follow-up time with a small number of missed patients. In this population, the expression of MCT1, MCT4, and CD147 was lower than that observed by Pinheiro et al. (19.4, 7.3 and 11.0%, respectively) [20]. GLUT1 and CAIX expressions were also lower than the frequencies of 46.0 and 18.0% seen in the study by Pinheiro et al. [17] and 28.5 and 12.5% in the study of Vleugel et al. [25]. It should be considered that in Pinheiro et al. studies [17, 20] and Vleugel et al. study [25], the percentage of the population with tumors larger than 5 cm ranged from 9.9 to 17.6%, while in the present study, tumor size was greater than 5.0 cm in 90.3% of the cases. In addition, the antibodies and the positivity criteria used by Vleugel et al. are different from those used in the present study [25].

In accordance with previous studies [17, 18, 20, 26], the expression of the metabolism-related proteins was associated with worse prognostic factors. For instance, tumor characteristics related to loss of differentiation and higher growth and probability of dissemination, like histological grade of Nottingham III, mitotic score 3 and nuclear grade G3 were associated with MCT1, GLUT1 and CAIX. In addition, presence of necrosis was associated with MCT4, GLUT1 and CAIX, while lymph node involvement was associated with MCT4, CD147 and GLUT1 expressions. Finally, the lack of ER and PR expression was associated with MCT1, CD147, CAIX and GLUT1. The hyperglycolytic and acid-resistant phenotype in undifferentiated cells is responsible for the acidification of the extracellular environment, which, in turn, stimulates tumor progression and dissemination [15, 27–30]. Also, rapid growth, partly maintained by the hyperglycolytic phenotype, leads to hypoxia and increased necrosis, which also contributes to the metabolic reprogramming towards an hyperglycolytic metabolism, thus creating a cyclic process to stimulate tumor growth and dissemination [15, 27–30]. Therefore, there would be a process of natural selection where tumor cells with characteristics of greater aggressiveness, when manifesting the hyperglycolytic phenotype, would have adaptive advantages for greater proliferation and dissemination.

The percentage of pCR observed (16.3%) is consistent with data seen in prospective phase II and III clinical trials, ranging from 15 to 30% and using sequential use of docetaxel to chemotherapy [31, 32] or weekly paclitaxel [33]. However, pCR is often related to higher survivals and is more frequently associated with aggressive tumors [7–12, 34–36]. This behaviour has been referred to as the “triple negative paradox phenomenon” [37]. It may be related to the expression of proto-oncogenes and immune response regulatory genes, as well as the lack of an additional therapeutic option (eg hormone therapy), which would allow the rapid evolution of the disease in those cases that do not reach pCR with NAC [37, 38]. In this study, pCR was also associated to aggressive tumors, occurring in 19.4% of triple negative compared to 9.1% in luminal A. Our results is in agreement with previous report describing pCR rates ranging from 20.0 to 34.0% in triple negative, and 0.0 to 7.5% in luminal A tumors [12]. Additionally, associations were observed between pCR and age, absence of ER expression, HER2 overexpression, mitotic score, as well as GLUT1 and CAIX expression. In multivariate analysis, only regional lymph nodes staging (TNM - N), mitotic score and CAIX expression were independent predictors of pCR.

To the best of our knowledge, CAIX expression has not been previously described as an independent predictor of pCR. Aomatsu et al. observed that CAIX expression is related to lower pCR rate and considered this protein a chemoresistance marker [39]. In that study, CAIX expression frequency was 46.0% [39], whereas in the present study it was only 7.4%. Another difference between the two studies is the frequency of pCR seen in 29.0% of patients in Aomatsu study versus 16.3% in the present one [39]. However, the differences in samples’ characteristics should be emphasized; while in the present study the sample was comprised of patients with locally advanced tumor treated with AC-T, the Aomatsu et al. study sample consisted of 102 patients with early-stage breast cancer treated with 5-fluorouracil, epirubicin, and cyclophosphamide [39].

Other explanations related to the phenotypic manifestation could explain the unprecedented result of the present study. In a recent study, Euceda et al. [40] evaluated, through magnetic resonance spectroscopy, the metabolic behavior of breast cancer of 122 patients treated with NAC and randomized to sequential use of bevacizumab. Good responders presented an initial metabolic profile related to greater aggressiveness and elevated levels of lactate were observed, which progressively increased throughout the treatment. The authors suggested that patients with tumors with a metabolic profile associated with increased aggressiveness are more likely to benefit from this treatment in terms of reduced tumor size, possibly due to a change in their phenotype - becoming metabolically non-glycolytic - or related to morphological changes that would block lactate excretion [40]. This would likely alter the tumor microenvironment, reducing extracellular acidity, which would improve the efficacy of chemotherapeutics, classified as weak bases that ionize under low pH conditions [41]. This context is very similar to that observed in the present study, especially with regard to the greater CAIX expression in pre-treatment tumors from patients who reached pCR after NAC. Even with the expression of a protein responsible for pH control and promoter of an appropriate microenvironment to tumor growth and proliferation, the expected aggressive phenotype was not able to manifest in the group of patients evaluated in this study, which allowed higher rates of pCR, contrary to the initial expectations.

In line with the association with pCR, CAIX expression was also associated with higher DFS and DSS. These findings were also not previously described, and go against previous studies showing CAIX as a poor prognostic factor [17, 39, 42, 43]. Generali et al. demonstrated women with breast cancer treated with epirubicin and tamoxifen had lower DFS and OS when expressing CAIX [42]. Similarly, Pinheiro et al. observed that CAIX expression was associated with an increased risk of relapse [17]. In the study by Aomatsu et al., in which CAIX expression was evaluated in breast cancer tumor samples before and after NAC, the presence of the protein was prognostic of lower DFS in both situations [39]. As a counterpoint, it is important to cite two studies. In the first one, Ivanova et al. evaluated breast cancer samples of 3455 patients and observed high expression of CAIX mRNA was associated with lower DFS in basal-like and triple negative subtypes and lower OS in luminal B, but not in luminal A and HER2 + [43]. On the other, Chen et al. evaluated the expression of CAIX and CAXII mRNA, enzymes with the same catalytic function, but with related different prognostics predictions (CAIX related to worse and CAXII to good prognosis) [44, 45]. Chen et al. observed high expression of CAIX mRNA was associated with increased survival in the luminal subtype while CAXII mRNA expression was linked to reduced survival in basal and HER2 positive breast cancer [44]. Furthermore, they suggest that CA enzymes could have their functions regulated by changes in the pH of the tumoral microenvironment [44]. Thus, we can assume that in our study, the conditions of the tumor microenvironment (related to the large tumor size and NAC based on AC-T) may have determined CAIX functional alterations and, consequently, may have been associated with pCR and higher survival. Moreover, in the samples evaluated in our study, the low CAIX expression could be compensated by a higher CAXII expression, unfortunately not evaluated by us. It should be noted the lack of correlation of triple-negative cases with pCR rates in the multivariate analysis. We consider, however, that this finding is strictly related to statistical power. Due to the number of included variables, the final sample size in this analysis was substantially reduced, probably determining this lack of correlation. In addition, among the triple-negative cases that demonstrated pCR, only one of them had CAIX expression. Given these data, we can state that there is no strong correlation between CAIX and pCR expression between triple-negative tumors, even with the result found in the multivariate analysis.

Since the biological material used in TMA construction is dated from 2005 to 2011, its quality should be considered as a limitation of this study. Although all the samples come from the same service, differences in the techniques of fixing and preserving the material should be considered, which could contribute to the reduction of antigenicity, decrease in the sensitivity of the IHC reaction and, of course, lower detection of protein expression [46, 47]. It is also worth noting that the TMA blocks used in the present study were composed of single samples from each patient and, as already mentioned, there were a considerable number of cases excluded by the lack of tumor representativeness.

## Conclusion

In this study, we describe for the first time CAIX expression as a predictor of pCR and its association with higher DFS and DSS in patients with locally advanced breast cancer treated by NAC using AC-T. Considering the size of the cohort and the long follow-up time, we believe these results give an important contribution to the knowledge about the participation of glycolytic metabolism to breast cancer response to chemotherapy. New studies evaluating other metabolic parameters such as expression of additional metabolism-related proteins, levels of metabolic byproducts and modifications in metabolism-related genes, could better clarify how the metabolic adaptations of cancer cells may be implicated in tumor behavior against certain therapies, as well as determine prognostic markers and new therapeutic targets within an ideal of personalized medicine.

## Supplementary information

**Additional file 1: Table S1.** Association between metabolism-related proteins expression and clinicopathologic characteristics. Table showing the association between metabolism-related proteins expression and clinicopathologic characteristics.

**Additional file 2: Table S2.** Association of clinicopathologic characteristics and proteins related to glycolytic metabolism with DFS, DSS and OS after NAC – Cox proportional hazards regression model. Table showing the association between clinicopathologic characteristics and proteins related to glycolytic metabolism with DFS, DSS and OS after NAC.

## Data Availability

The datasets used and/or analyzed during the current study are available from the corresponding author on reasonable request.

## Abbreviations

AC: Doxorubicin and cyclophosphamide
BC: Breast cancer
CAIX: Carbonic anhydrase IX
DFS: Disease-free survival
DSS: Disease-specific survival
GLUT1: Glucose transporter-1
MCT: Monocarboxylate transporters
NAC: Neoadjuvant chemotherapy
NSABP: National Surgical Adjuvant Breast and Bowel Project
OS: Overall survival
pCR: Pathological complete response
T: Paclitaxel
TMA: Tissue microarray
